# Antimalarial Activity of Hydromethanolic Crude Extract and Chloroform Fraction of *Brucea antidysenterica* Leaves in *Plasmodium berghei*-Infected Mice

**DOI:** 10.1155/2021/2089114

**Published:** 2021-10-13

**Authors:** Tezera Jemere Aragaw, Kefyalew Ayalew Getahun

**Affiliations:** Department of Pharmacology, College of Medicine and Health Sciences, University of Gondar, Gondar, Ethiopia

## Abstract

**Background:**

Different parts of *Brucea antidysenterica* are used in traditional and alternative medicine in Ethiopia for the treatment of different health problems including malaria and have good *in vitro* antimalarial activity. However, no in vivo study was conducted to substantiate the claim. Our study planned to determine the antimalarial effect of *B. antidysenterica* extract.

**Methods:**

Swiss albino mice (6–8 weeks old, 20–28 g) were inoculated with *Plasmodium berghei*. Different doses of both hydromethanolic extract and chloroform fraction were orally given at 100, 200, and 400 mg/kg/day.

**Results:**

The parasitemia suppression percent of hydromethanolic crude extract and chloroform fraction in chemosuppressive tests ranged between 33.48 and 75.93% and 38.32 and 76.64%, respectively. The hydromethanolic crude extract and chloroform fraction exhibited the curative effect of 46.75–70.91% and 50.30–80.06% parasitemia suppression, respectively (*p* < 0.001), compared with negative control.

**Conclusion:**

From our study, it is concluded that the hydromethanolic crude extract and chloroform fraction of *B. antidysenterica* leaves showed promising antiplasmodial effects against *Plasmodium berghei*. This upholds the folkloric use of *B. antidysenterica* leaves and the thought of as a possible source to develop new antimalarial agents.

## 1. Background

There were approximately 3.3 billion people globally in danger of malaria and 219 million malaria cases and 435,000 deaths worldwide in 2017, and the quantity of cases and burdens increased in Africa [1]. Approximately 125 million pregnant women in 2017 were in danger of infection [2]. 200 thousand yearly infant deaths are caused by *Plasmodium falciparum* resistance to chloroquine and sulfadoxine-pyrimethamine [3]. In Africa, children below five years old who have at least six malaria-associated illnesses annually are chronic victims. After they are fatally afflicted, children who develop severe symptoms often die within 72 hours. Malaria parasites that drain vital nutrients and impair physical and intellectual development are the principal reasons for poor school attendance of youngsters who survive [4]. In Ethiopia, 75% of the land below 2000 meters is malarious with 68% people in danger from infection, with a mean of 5 million cases a year with increased health service expenses and low productivity [5]. In Ethiopia, malaria is among the ten top leading causes of outpatient visit, hospital admission, morbidity, and mortality in children under the age of 5 and adults [6]. *Plasmodium falciparum* resistance to chloroquine and sulfadoxine/pyrimethamine has been an enormous setback in the fight against malaria [7]. In Ethiopia, 80% of the people and 90% of livestock traditional medicines served as an option as modern services are either limited or unavailable [8]. For *in vivo* evaluation of antimalarial compounds, animal models such as primates, avians, and rodents are used [9]. The choice depends upon the breadth of the response, practical consideration, sensitivity, reproducibility, technical complexity, the quantity of the test compound needed, and price per test, even though this model is not entirely extrapolating the results to humans [10].

Among the extensively used animal models of malaria, mice are ideal for *in vivo* tests. They are small (20–30 g), friendly, and easy to manipulate [11]. Extracts that show an adequate or above 50% malarial *in vivo* parasitemia suppression at doses of 500, 250, and 100 mg/kg/day are often categorized as moderate, good, and excellent, respectively [12].

*In vivo* antimalarial screening results of percent parasitemia inhibition of hydromethanolic extracts of various traditionally used plants and their parts in a four-day suppressive test were as follows: 100–400 mg/kg/day extract dose of *Annona senegalensis* leaves (57.1–76.3%) [13], *Aloe debrana* leaves (30.21–44.15%), *Dodonaea angustifolia* leaves (57.74–71.51%), *Clerodendrum myricoides* leaves (54.14–65.95%) [14], *Carica papaya* fruit rinds (8.18–18.39%) and roots (10.31–25.63%) [15], *Gardenia ternifolia* root bark (32.58–47.02%) [16], *Croton macrostachyus* leaves (44–78%) [17], *Sphenocentrum jollyanum* leaves (74.75% at 200 mg/kg/day) [18], *Justicia schimperiana* leaves (64.98–81.49%) [19], *Strychnos mitis* leaves (36.56% at 200 mg/kg day) [20], *Piper betle* leaves (52.94–82.31%) [21], *Croton zambesicus* leaves (70.7–80.7%) [22], and *Napoleona imperialis* roots (96.88–99.1%) [23].

*Brucea antidysenterica* is a monoecious shrub up to 7–15 meters tall, with alternate, heart-shaped, gray or brown color leaf-scars; young stems or twigs have red or brown hairs. Fruits have up to 4 ellipsoid mericarps with one seed per mericarp [24].

*Brucea antidysenterica* roots, fruits, and bark are accustomed for the treatment of fever, helminthic infections, and dysentery. The boiled roots, leaves, seeds, fruits, and bark are accustomed as a remedy for indigestion, stomachache, and diarrhea. To relieve asthma, the roots and leaves are cooked with meat and used. The twigs and leaves are prepared with butter or fruit (ripe) with honey to treat leprosy and scrofula. Cancerous skin tumors and sexually transmitted diseases are treated with leaves and roots, respectively. The colic and bloating in cattle are relieved by powdered leaves. *B. antidysenterica* root extracts are used to treat rabies and also used as fire wood, leaves serve as animal feed, and the wood is used for house construction [25–27].

The antimalarial activity of an extract showing an IC50 value of ≤5 *μ*g/ml was classified as high, whereas extracts with IC_50_ values between 5 *μ*g/ml and 10 *μ*g/ml, 10 *μ*g/ml and 50 *μ*g/ml, and above 50 *μ*g/ml were considered moderate, low, and inactive, respectively [28]. The activity of bruceantin obtained from the leaves and stem bark of *B. antidysenterica* induces apoptosis involving the caspase and mitochondrial pathways of myeloma cell lines, lymphoma, and leukemia [29, 30].

Bruceantin and simalikalactone D, obtained from *B. antidysenterica*, showed IC_50_ values of 0.0008 and 0.0009 *μ*g/ml against *Plasmodium falciparum* and (IC_50_ of bruceantin = 0.018 *μ*g/ml) *Entamoeba histolytica* [31, 32].

The hydromethanolic crude extract obtained from *B. antidysenterica* leaves showed a high *in vitro* activity, which helps carry on *in vivo* study to determine whether the hydromethanolic crude extract and chloroform fraction have antimalarial activities using different parameters. From the *in vivo* antimalarial study, extracts up to a dose of 1000 mg/kg exhibited greater than or equal to 30% parasitemia suppression compared with the negative control and hence are considered active [33].

### 1.1. Rationale of the Study

Emergence of resistance of *Plasmodium falciparum* to chloroquine and sulfadoxine-pyrimethamine causes morbidity and mortality in all segments of the population and is related to enormous setback in the fight against malaria [4–7]. So, there is a desire to possess a new effective agent. Ethnobotanical studies of *B. antidysenterica* showed that its roots, fruits, and bark are accustomed for the treatment of fever, helminthic infections, and dysentery. The boiled roots, leaves, seeds, fruits, and bark are accustomed as a remedy for indigestion, stomachache, and diarrhea. To alleviate asthma, the roots and leaves are cooked with meat and used. The twigs and leaves are prepared with butter or fruit (ripe) with honey to treat leprosy and scrofula. Cancerous skin tumors and sexually transmitted diseases are treated with leaves and roots, respectively. The colic and bloating in cattle are relieved by powdered leaves. Its roots are used to treat rabies and also used as an energy source, and its wood is utilized for house construction [25–27]. The study of secondary metabolites of the hydromethanolic crude extract of *B. antidysenterica* leaves showed a high *in vitro* antimalarial activity, which helps hold on *in vivo* study to see whether the hydromethanolic crude extract and chloroform fraction have antimalarial activities [31, 32].

No report is obtainable within the literature suggesting whether the leaves possess *in vivo* antimalarial activity. This study was therefore planned to evaluate the hydromethanolic crude extract and chloroform fraction of *B. antidysenterica* leaves for antimalarial activity in *P. berghei*-infected mice and additionally acute oral toxicity in the Ethiopian folk medicine.

## 2. Materials and Methods

### 2.1. Drugs, Chemicals, Supplies, and Equipment

Chloroquine phosphate (CADILA Pharmaceuticals PLC, Ethiopia), absolute methanol (LOBA Chem. Ltd, India), ammonia (Blulux Laboratories (P) Ltd, India), benzene and chloroform (SDFCL Fine Chem. Ltd, India), concentrated sulfuric acid (HiMedia Laboratories Pvt. Ltd, India), distilled water, emersion oil, and absolute ethyl alcohol (GMC Chemical Manufacturing, Ethiopia), ferric chloride and Giemsa stain (AppliChem, Germany), glacial acetic acid, n-hexane, and sodium chloride 0.9% IV infusion (Sansheng Pharma, Ethiopia), trisodium citrate (3.8%), Wagner's and Mayer's reagent, aluminum foil, disposable glove (medium size), Gauze 40 mesh, and heparinized syringes with needle of 5/10 ml (Jiangsu Kanghua Medical Equipment Co. Ltd, China), insulin syringes 1 ml (Changzhou Jinlong Medical Plastic Appliance Co. Ltd, China), microscopic slide frosted (1 mm–1.2 mm thick and 25.4 mm × 76.2 mm), Whatman filter paper (15 cm diameter and 0.1 *μ*m pore diameter), beakers, lyophilizer, dry oven (250 ± 10% volts AC, 600 watts, 50/60 Hz), electrical balance, funnels, HemoCue 3001 machine, HemoCue cuvette, light microscope, measuring cylinder, mice cage, mice gavage, pasture pipette, separating funnel, and stainless scissor 14 cm long.

### 2.2. Plant Material

*Brucea antidysenterica* fresh leaves were collected on May 13, 2019, from Agew Awi Zone within Amhara Region. It is located at 10°57′N and 36°56′E in Banja Shekudad District at an elevation of 2560 meters above sea level. The collected leaves were wrapped and covered with plastic sheets during transportation. The specimen of the plant was authenticated as *Brucea antidysenterica* by a botanist, within the Department of Biology, the University of Gondar, and was deposited within the herbarium with a voucher specimen No: 005/KAG/2020 for future reference.

### 2.3. Preparations of Crude Methanolic Extract

*Brucea antidysenterica* leaves were dried in shadow and at an ambient temperature, reduced in size by hand compression, and stored at room temperature until the extraction. *Brucea antidysenterica* leaf powder of 400 g was weighed with an electrical balance and transferred to a beaker, and 2400 ml of 80% hydromethanolic solution was added and shaken in between to homogenize. After three days of maceration, extraction was performed using thick layers of 40 mesh gauze and filtered with Whatman paper № 1 twofold, and the 2^nd^ extraction was performed again after three days post maceration; the 3^rd^ extraction was repeated another 72 hours later (an entire of nine days). The filtrates were combined and were frozen overnight using a deep freezer and freeze-dried in a lyophilizer at −50°C to eliminate water. The yield was measured and calculated to be 42.6 g (10.65%) and stored in a refrigerator at 4°C until use [34, 35].

### 2.4. Solvent Fractionation of Crude Extract

Hydromethanolic crude extract of *B. antidysenterica* leaves was processed for further fractionation using polar and nonpolar solvents with increasing polarity n-hexane (0.1), chloroform (4.1), and water (10.2). Dried hydromethanolic crude extract of *B. antidysenterica* leaves of 70 gm was weighed and soaked in 420 ml distilled water and was gently shaken to combine. The mixture was transferred to a separatory funnel. Then, equal volume of n-hexane was added to it. After being gently shaken, the extract was allowed to settle and separated into two distinct layers consistent with their density. The upper n-hexane layer was collected, and then the same procedure was repeated 3 times. After the gathering of n-hexane fraction of the extract, the water was fractionated with chloroform 3 times with same procedure of n-hexane and also the bottom chloroform layer was collected, leaving the upper aqueous fraction. Finally, the aqueous fraction was collected. The filtrates of chloroform and n-hexane fractions were concentrated using a rotary evaporator and dried using a dry oven at 40°C. The aqueous fraction was frozen in a refrigerator overnight and was dried using a lyophilizer. The percentage yield was calculated, and the yield was stored at 4^o^C until use [36].

### 2.5. Phytochemical Screening

The qualitative phytochemical screening tests of secondary metabolites were performed on 80% hydromethanolic crude extract of *Brucea antidysenterica* leaves using standard chemicals and procedures that were utilized in previous research [37–47].

### 2.6. Animals and Parasite

We purchased mice (Swiss albino) aged 6–8 weeks weighing 20−28 g, either sex, from the Ethiopian Public Health Institute (EPHI), Addis Ababa. The mice were kept (five to 6 mice/cage) in clean polyethylene plastic cages with a wire mesh top containing a hygienic bed in fact sawdust (regularly changed every 3 days) and retained in a well-ventilated room 24–25°C, 50–60% humidity, and a light-dark cycle of 12 hours with free delivery of ordinary pellet diet purchased from local suppliers and clean potable tap water. Then, the mice were acclimatized with the test environment for seven days before the initiation of the experiment. The care and handling of mice were performed with globally accepted standard laboratory protocols and guidelines [35, 48, 49]. The research was performed as per the agreement of the ethical clearance document Ref. No: DU/RPD/102/2015.

Chloroquine-sensitive *Plasmodium berghei* was obtained from the Traditional Medicine Research Department, EPHI, in Addis Ababa and transported by infecting the donor mice and maintained the parasite until the actual procedure of the study.

### 2.7. Acute Toxicity Test

Five female Swiss albino mice were kept for seven days before dosing to acclimatize to the test environment. One mouse was randomly taken to perform preliminary toxicity observation on free access to potable tap water but fasted for four hours and weighed, and then hydromethanolic crude extract of 2 g/kg leaves of *B. antidysenterica* was administered via the oral route. Firm inspection was done for half an hour and periodically for the primary 24 hours, for consecutive fourteen days. Observation was majorly focused on changes in skin and fur, eyes, mucous membranes, respiratory, circulatory, autonomic, and central nervous system, and somatomotor activity and behavior patterns were observed. Tremors, convulsions, salivation, diarrhea, lethargy, sleep, and coma were evaluated. The mouse did not show any sign of toxicity for four days in initial toxicity inspection. The remaining four Swiss albino female mice were dosed by similar doses and followed up for 14 days [35, 48, 50].

### 2.8. Pharmacologic Screening (4-Day Suppressive Test)

The evaluation of crude hydromethanolic extracts and chloroform fraction of *B. antidysenterica* leaves for *in vivo* antimalarial activity on rodent protozoan *P. berghei* was performed. Donor *P. berghei*-infected Swiss albino mice (parasitemia of roughly 30%) were sacrificed by decapitation; then blood was drawn from the heart by cardiac puncture with a disposable sterile syringe and needle. Sterile 0.9% normal saline and anticoagulant trisodium citrate were used to dilute the blood; 0.2 ml of blood contained about 10^7^ infected erythrocytes, and the mice were infected by 0.2 ml blood suspension intraperitoneally to cause consistent infection in mice [49]. Randomly divided the mice in groups of eight, six mice in each group, free access to food and water, and weighed. The doses of crude hydromethanolic extract and fraction of chloroform of *B. antidysenterica* leaves were adjusted from the safest dose of acute toxicity study (2000 mg/kg), and the doses were 20% (400 mg/kg/day), 10% (200 mg/kg/day), and 5% (100 mg/kg/day) from higher to lower doses, respectively. Three different doses of hydromethanolic crude extract were administered to the mice for 4 days, and they were grouped accordingly: Group I, 100 mg/kg/day; Group II, 200 mg/kg/day, and Group III, 400 mg/kg/day; and similarly, mice were grouped according to the chloroform fraction: Group IV, 100 mg/kg/day, Group V, 200 mg/kg/day), and Group VI, 400 mg/kg/day. Group VII received chloroquine base 10 mg/kg/day (positive control), and Group VIII received a solvent (10 ml/kg/day) composed of Tween 80 (7 ml) + ethanol 96% (3 ml) + distilled water (90 ml) (negative control) [17, 35, 51] orally using oral gavage after three hours of parasite inoculation.

### 2.9. Rane's (Curative) Test

Evaluations of crude hydromethanolic extract and chloroform fraction of *B. antidysenterica* leaves were performed with the strategy described by curative methods [9]. About 10^7^ infected erythrocytes were inoculated in mice intraperitoneally on day 0 and randomly divided into eight groups, six mice in each group. Group I (negative control) treated with solvent 10 ml/kg/day, Group II treated with crude hydromethanolic extract at 100 mg/kg/day, Group III treated with crude hydromethanolic extract at 200 mg/kg/day, Group IV treated with crude hydromethanolic extract at 400 mg/kg/day, Group V treated with chloroform fraction at 100 mg/kg/day, Group VI treated with chloroform fraction at 200 mg/kg/day, Group VII treated with chloroform fraction at 400 mg/kg/day, Group VIII treated with chloroquine base at 10 mg/kg/day. Mice were weighed and maintained on a pellet diet. Administration of the crude hydromethanolic extract at 100, 200, and 400 mg/kg/day, chloroform fraction at 100, 200, and 400 mg/kg/day, chloroquine base at 10 mg/kg/day, and a solvent (10 ml/kg) prepared from Tween 80 (7 ml) + ethanol 96% (3 ml) + distilled water (90 ml) to the respective groups was started on third day and continued once daily for five days. A Giemsa-stained thin blood film was prepared from the tail of each mouse daily for five days (day 3, 4, 5, 6, and 7) to quantify the parasitemia level. The Swiss albino mice were followed up for 30 days and calculated arithmetically to determine the mean survival time for each group starting from the date of infection for 30 days (D0–D29) [17, 35].

#### 2.9.1. Determination of Parasitemia

Starting from infection at 96 hours, a drop of blood was collected from the mice by the vein section of the tail and transferred onto to a microscopic slide and drawn evenly across the second slide to create a thin blood film and allowed to dry at room temperature, fixed with methanol, and stained with 10% Giemsa stain for half an hour. Slides were viewed using light microscopy with oil immersion (1000x magnification). Parasite load in percent was determined by counting parasitized red blood cells out of 200 RBCs in random fields of the microscope. For each mouse, five fields were examined. Then, parasitemia percent was calculated by the following formula [17, 35]:

(1) $$\begin{array}{c} \%\text{parasitemia}=\frac{\text{total number of PRBC}}{\text{total number of RBC}}\times 100, \end{array}$$

where PRBC represents the parasitized red blood cells and RBC means red blood cells.

Average percentage of parasitemia suppression was calculated as follows:

(2) $$\begin{array}{c} \text{average \% of parasitemia supression}=\frac{\text{avg. \% of parasitemia in negative control}-\text{avg. \% of parasitemia in test}}{\text{avg. }\%\text{ of parasitemia in negative control}}\times 100, \end{array}$$

where Av = average.

#### 2.9.2. Determination of Body Weight

The body weight of the mice was measured to judge whether the test extract of *B. antidysenterica* leaves prevented weight loss. The weight was assessed on day 0 (after an infection was initiated) and on day 4 (96 hours) post infection [35, 52].

(3) $$\begin{array}{c} \text{average \% body weight loss}=\frac{\text{avg. body weight of mice at day 0}-\text{avg. body weight of mice at day }4\;\left(\text{g}\right)}{\text{avg. body weight of mice at day 0 }\left(\text{g}\right)}\times 100. \end{array}$$

#### 2.9.3. Determination of Hemoglobin Level

The hemoglobin level of the mice was measured to judge the effectiveness of hydromethanolic crude extract and chloroform fraction of *Brucea antidysenterica* leaves in preventing anemia. Hemoglobin was evaluated by using a hemoglobin cuvette and hemoglobin machine. Blood samples were collected from the vein section of mice's tail by a trained medical laboratory technologist with optimum pressure applied on the tail and filled in a microcuvette (Hb 301) approximately 10 *μ*l. Excess blood was removed before inserting the microcuvette into the machine. Then, hemoglobin levels in g/dl were displayed automatically, and the mean hemoglobin level was determined using the following formula [35, 53]:

(4) $$\begin{array}{c} \text{mean hemoglobin}=\frac{\text{sum of hemoglobin for all mice in a group}\left(\text{ in }\text{g}/\text{dl}\right)}{\text{total number of mice in that group}}. \end{array}$$

#### 2.9.4. Determination of Mean Survival Time

The Swiss albino mice were maintained with free delivery of ordinary pellet diet purchased from local suppliers and clean potable tap water. For 28 days, the mice were observed and deaths were recorded to judge the crude hydromethanolic extract and chloroform fraction effect for improvement in survival days [9].

(5) $$\begin{array}{c} \text{Mean survival times}=\frac{\text{Sum of survival times for all mice a group}\left(\text{in days}\right)}{\text{Total number of mice in that group}}. \end{array}$$

#### 2.9.5. Data Analysis

The results of the study were expressed as mean ± standard error of the mean (M ± SEM). Parasitemia comparison and statistical significance were resolved by one-way ANOVA descriptive statistics. Post hoc tests for multiple comparisons of Tukey's HSD and paired *t*-tests were employed to check significance for the difference between initial and final results within and between identical groups using SPSS for Windows (version 20.0) IBM statistical package. All data were analyzed at a 95% confidence interval, and *p* < 0.05 was considered statistically significant [54].

## 3. Results

### 3.1. Phytochemical Screening

The evaluation of phytoconstituents of crude hydromethanolic extract of *B. antidysenterica* leaves indicated existence of sterols, alkaloids, phenols, flavonoids, saponins, terpenoids, and tannins, but alkaloids were only present in chloroform fraction of *B. antidysenterica* leaves (see Table 1).

### 3.2. Evaluation of Acute Oral Toxicity

The evaluation of acute oral toxicity did not show any physical or behavioral changes or deaths up to 14 days from the administration of crude hydromethanolic extract at 2 g/kg.

### 3.3. Antimalarial Suppressive Test

The antimalarial suppression evaluation of crude hydromethanolic extract and chloroform fraction of *B. antidysenterica* leaves in *P. berghei*-infected mice showed a lower parasite level compared with their respective solvent-treated mice. The parasite was totally cleared in mice treated with chloroquine base 10 mg/kg. The crude hydromethanolic extract of *B. antidysenterica* leaves at 100, 200, and 400 mg/kg/day showed 33.48, 58.36, and 75.93% parasitemia suppression, respectively, whereas the chloroform fraction of *B. antidysenterica* leaves at 100, 200, and 400 mg/kg/day showed 38.32, 64.49, and 76.64% parasitemia suppression, respectively; therefore, the differences in the results were highly significant (*p* < 0.001) when compared with solvent-treated mice at day 4 (see Table 2).

### 3.4. Effects of Crude Hydromethanolic Extract and Chloroform Fraction of *B. antidysenterica* Leaves on Body Weight in *P. berghei*-Infected Mice

*P. berghei*-infected mice treated with crude hydromethanolic extract of *B. antidysenterica* leaves at 100 mg/kg lost 9.34 ± 1.61% (*p* = 0.770) of weight, 200 mg/kg 6.49 ± 1.19% (*p* = 0.844) of weight, and 400 mg/kg/day 1.78 ± 0.98% (*p* < 0.001) of weight. Chloroform fraction of *B. antidysenterica* leaves at 100 mg/kg lost 9.24 ± 1.62% (*p* = 0.741) of weight, 200 mg/kg 5.43 ± 0.95% (*p* = 0.023) of weight, and 400 mg/kg/day 0.18 ± 0.76% (*p* < 0.001) of weight. Chloroquine base at 10 mg/kg/day gained 4.10 ± 1.23% (*p* < 0.001) of weight and mice treated with solvent lost 12.49 ± 2.38% of weight (see Figure 1).

### 3.5. Activity of Crude Hydromethanolic Extracts and Chloroform Fraction of *B. antidysenterica* Leaves on Average Hemoglobin Level of *P. bergei*-Infected Mice

The average hemoglobin level after administration of crude hydromethanolic extract of *B. antidysenterica* leaves at 100 mg/kg/day was 8.07 ± 0.23 g/dl (*p* = 0.251), 200 mg/kg/day 9.87 ± 0.40 g/dl (*p* < 0.001), and 400 mg/kg/day 12.95 ± 0.54 g/dl (*p* < 0.001); for chloroform fraction at 100 mg/kg/day was 9.38 ± 0.30 g/dl (*p* < 0.001), 200 mg/kg/day 11.75 ± 0.32 g/dl (*p* < 0.001), and 400 mg/kg/day 13.52 ± 0.38 g/dl (*p* < 0.001); for chloroquine base at 10 mg/kg/day was 14.15 ± 0.32 g/dl (*p* < 0.001); and for noninfected mice was 14.37 ± 0.24 g/dl (*p* < 0.001) compared with the negative control (6.55 ± 0.68) (see Figure 2).

### 3.6. Effects of Crude Hydromethanolic Extract and Chloroform Fraction of *B. antidysenterica* Leaves on Mean Survival Time of *P. bergei*-Infected Mice in a 4-Day Suppressive Test

Hydromethanolic crude extract of *B. antidysenterica* leaves at 100, 200, and 400 mg/kg/day showed mean survival time of 6.5 ± 0.43 days (*p* = 0.849), 7.67 ± 0.42 days (*p* = 0.0.218), and 12.67 ± 0.76 days (*p* < 0.001), and chloroquine base at 10 mg/kg/day showed 23 ± 1.18 (*p* < 0.001) days, respectively. Chloroform fraction of *B. antidysenterica* leaves at 100, 200, 400 mg/kg/day showed 7.9 ± 0.36 (*p* = 0.070), 9.45 ± 0.33 (*p* = 0.001), and 14.67 ± 0.33 days (*p* < 0.001) of mean survival time, and chloroquine base at 10 mg/kg/day showed 23 ± 1.18 (*p* < 0.001) days, respectively, and the mice treated with solvent showed 5.5 ± 0.34 days (see Figure 3).

### 3.7. Antimalarial Curative Test

The antimalarial curative test of hydromethanolic crude extract of *B. antidysenterica* leaves at 100, 200 (62.11%), and 400 mg/kg showed 46.75%, 62.11%, and 70.91% parasitemia inhibition, respectively; chloroform fraction at 100, 200, and 400 mg/kg showed 50.3%, 65.5%, and 80.06% parasitemia inhibition, respectively; and chloroquine base at 10 mg/kg showed 93.13% parasitemia inhibition in *P. berghei*-infected mice at day 5; therefore, the differences in the results were highly significant (*p* < 0.001) when compared with the negative control (see Table 3).

The hydromethanolic crude extract of *B. antidysenterica* leaves at 100, 200, and 400 mg/kg exhibited 7.50 ± 0.43, 9.33 ± 0.33, and 12.17 ± 0.60 days of mean survival time, respectively; chloroform fraction of *B. antidysenterica* leaves at 100, 200, and 400 mg/kg showed 9.50 ± 0.43, 12.33 ± 0.42 days, and 15.33 ± 0.76 days of mean survival time, respectively; and chloroquine base at 10 mg/kg/day showed a mean survival time of 30.00 ± 0.00 days in the curative test; therefore, the differences in the results were highly significant (*p* < 0.001) when compared with negative control (5.33 ± 0.21 days) (see Table 3).

### 3.8. Effects of Crude Hydromethanolic Extract and Chloroform Fraction of *B. antidysenterica* Leaves on Mean Survival Time of Mice Infected with *P. bergei* in a Curative Test

Hydromethanolic crude extract of *B. antidysenterica* leaves at 100, 200, and 400 mg/kg/day showed 7.50 ± 0.43 (*p* = 0.003), 9.33 ± 0.33 (*p* < 0.001), and 12.17 ± 0.60 (*p* < 0.001), respectively, and chloroquine base at 10 mg/kg/day showed 30.00 ± 0.00 (*p* < 0.001) days of mean survival time in a curative test. Chloroform fraction of *B. antidysenterica* leaves at 100, 200, and 400 mg/kg/day showed 9.50 ± 0.43 (*p* = 0.070), 12.33 ± 0.42 (*p* = 0.001), and 15.33 ± 0.76 (*p* < 0.001), respectively, and chloroquine base at 10 mg/kg/day showed 30.00 ± 0.00 (*p* < 0.001) days of mean survival time in a curative test; and mice treated with solvent showed 5.33 ± 0.21 days (see Figure 4).

## 4. Discussion

Resistance of *Plasmodium falciparum* to chloroquine and sulfadoxine-pyrimethamine causes morbidity and mortality in all segments of the population and is associated with enormous setback in the fight against malaria [4–7]. There is a need to have a new effective agent. Therefore, we assessed the antimalarial activity of hydromethanolic crude extract and chloroform fraction of *B. antidysenterica* leaves in *P. berghei*-infected mice. Ethnobotanical studies of *B. antidysenterica* roots, fruits, and bark are accustomed for the treatment of fever, helminthic infections, and dysentery. The boiled roots, leaves, seeds, fruits, and bark are accustomed as a remedy for indigestion, stomachache, and diarrhea. To relieve asthma, the roots and leaves are cooked with meat and used. The twigs and leaves are prepared with butter or fruit (ripe) with honey to treat leprosy and scrofula. Cancerous skin tumors and sexually transmitted diseases are treated with leaves and roots, respectively. The colic and bloating in cattle are relieved by powdered leaves. Its roots are used to treat rabies and also used as an energy source, and the wood is used for house construction [25–27]. The study of secondary metabolites of hydromethanolic crude extract of *B. antidysenterica* leaves showed a high *in vitro* activity, which helps carry on *in vivo* study to determine whether the hydromethanolic crude extract and chloroform fraction have antimalarial activities [31, 32]. *B. antidysenterica* contains considerable constituents of secondary bioactive constituents such as alkaloids, flavonoids, phenols, saponins, sterols, tannins, and terpenoids. The antimalarial effects of both hydromethanolic crude extract and chloroform fraction of *B. antidysenterica* leaves have higher mean percent parasitemia inhibition, reduction in weight, prevention of anemia, and a rise in mean survival time in days in a dose-dependent manner, which may be related to these secondary metabolites. Alkaloids have the capacity to DNA intercalation and terminate division of cells [40]. Flavonoids have the potential of complexing with soluble and intracellular proteins of cell components of organisms. Microbial membranes are at risk of being destroyed with flavonoids of high lipophilicity and inactivate toxins and inhibited isolated enzymes and complexing activities [40, 41]. Phenolic compounds produce inhibition of enzymes on oxidation and sulfhydryl interaction and other nonspecific proteins of microorganisms and produce toxicities [42]. Tannins have the power to initiate covalent, hydrogen, hydrophobic bonding, and complexing host-mediated tumor activity and phagocytosis [40]. The terpenes' mode of activity remains obscured, but compounds with this lipophilic character may disrupt membranes [40, 41]. These secondary metabolites present in *B. antidysenterica* leaves are going to be accustomed as a remedy for various ailments traditionally. Because of the presence of these secondary metabolites, *B. antidysenterica* has high healing potential, which is confirmed by the obtained results of the antimalarial activity.

The crude hydromethanolic extract did not produce toxicity and death at the test dose of the extract during the observation period. *B. antidysenterica* leaves hydromethanolic extract was nontoxic to tested mice and within the ranges tested during this study. Due to species variation, we cannot apply this finding to humans. Therefore, the crude hydromethanolic extract and chloroform fraction of *B. antidysenterica* leaves were administered in *Plasmodium berghei*-infected mice, which exhibited a dose-dependent activity in percent parasitemia inhibition. The crude hydromethanolic extract of *B. antidysenterica* leaves on a 4-day suppressive test on mice infected with *P. berghei* at 100 mg/kg/day showed an average percent parasitemia suppression (33.48%) higher than *Carica papaya* fruit rinds (8.18%) and roots (10.31%) [15] and less than *Annona senegalensis* leaves (57.1%) [13], *Justicia schimperiana* leaves (64.98%) and roots (49.51%) [19], *Piper betle* leaves (52.94%) [21], and *Croton zambesicus* leaves (70.7%) [22]. The crude hydromethanolic extract of *B. antidysenterica* leaves in an exceedingly 4-day suppressive test on mice infected with *P. berghei* at 200 mg/kg/day showed an average percent parasitemia suppression (58.36%) higher than *Clerodendrum myricoides* leaves (54.14%), *Dodonaea angustifolia* leaves (57.74%), *Aloe debrana* leaves (30.21%) [14], *Carica papaya* fruit rinds (17.16%) and roots (10.15%) [15], *Gardenia ternifolia* root bark (32.58%) [16], *Croton macrostachyus* leaves (44.00%) [17], *Sphenocentrum jollyanum* root (54.15%) [18], *Justicia schimperiana* leaves (37.1%) [19], and *Strychnos mitis* leaves (36.56%) [20] and less than *Annona senegalensis* leaves (59.3%) [13], *Sphenocentrum jollyanum* leaves (74.75) [18], *Piper betle* leaves (70.51%) [21], *Croton zambesicus* leaves (80.7%) [22], and *Napoleona imperialis* roots (99.1%) [23]. The crude hydromethanolic extract of *B. antidysenterica* leaves in an exceedingly 4-day suppressive test on mice infected with *P. berghei* at 400 mg/kg/day showed an average percent parasitemia suppression (75.93%) higher than *Clerodendrum myricoides* leaves (65.95%), *Dodonaea angustifolia* leaves (71.51), *Aloe debrana* leaves (44.15%) [14], *Carica papaya* fruit rinds (18.39) and roots (25.63%) [15], *Gardenia ternifolia* root bark (47.02%) [16] and less than *Annona senegalensis* leaves (76.3%) [13], *Croton macrostachyus* leaves (78%) [17], *Justicia schimperiana* leaves (81.49%) [19], *Piper betle* leaves (82.31%) [21], and *Napoleona imperialis* roots (96.88%) [23]. The chloroform fraction of *B. antidysenterica* leaves in an exceedingly 4-day suppressive test on mice infected with *P. berghei* at 100 mg/kg/day showed an average percent parasitemia suppression (38.32%) higher than *Carica papaya* fruit rinds (10.72%) and roots (9.77) [15] and *Strychnos mitis* leaves (26.84%) [20]. The chloroform fraction of *B. antidysenterica* leaves in a very 4-day suppressive test on mice infected with *P. berghei* at 200 mg/kg/day showed an average percent parasitemia suppression (64, 49%) higher than *Carica papaya* fruit rinds (24.2%) and roots (25.25) [15], *Gardenia ternifolia* root bark (24.51%) [16], *Croton macrostachyus* leaves (49.4%) [17], *Justicia schimperiana* leaves (16.4%) [19], and *Strychnos mitis* leaves (31.71%) [20]. The chloroform fraction of *B. antidysenterica* leaves during a 4-day suppressive test on mice infected with *P. berghei* at 400 mg/kg/day showed an average percent parasitemia suppression (76.64%) higher than *Carica papaya* fruit rinds (37.65%) and roots (48.11%) [15], *Gardenia ternifolia* root bark (31.13%) [16], *Croton macrostachyus* leaves (66.2%) [17], *Justicia schimperiana* leaves (26.32%) [19], and *Strychnos mitis* leaf (39.72%) [20].

Comparing the results obtained from this study, the crude hydromethanolic extract and chloroform fraction showed significant parasitemia inhibition compared with the mice treated with solvent. Extracts that show an adequate or above 50% proportion of malarial *in vivo* parasitemia inhibition at doses of 500, 250, and 100 mg/kg/day are often categorized as moderate, good, and excellent, respectively [12]. Supporting this classification, the hydromethanolic crude extract of *B. antidysenterica* leaves at 200 and 400 mg/kg/day showed 58.36 and 75.93% and chloroform fraction of *B. antidysenterica* leaves at 200 and 400 mg/kg/day showed 64.49% and 76.64% parasitemia suppression in *P. berghei*-infected mice, respectively, and therefore considered having good to moderate antiplasmodial activity. A more robust percentage of parasitemia inhibition was observed in chloroform fraction than the crude hydromethanolic extract on the identical doses. The results of our study indicated that the compounds extracted from *B. antidysenterica* leaves which have antimalarial activities were soluble in both hydromethanol and chloroform.

The crude hydromethanolic extract of *B. antidysenterica* leaves at 400 mg/kg/day prevented percent weight loss significantly compared with mice treated with solvent. The percent weight loss decreased in mice treated with both chloroform fraction and crude hydromethanolic extract from lower to higher doses. An increase in mean body weight was observed in mice treated with chloroquine base as shown in Figure 1. This can be attributed to the reduction in morbidity because of parasite clearance and their normal feeding.

The three different doses of both the chloroform fraction and crude hydromethanolic extract of *B. antidysenterica* leaves showed an increase in the hemoglobin level compared with mice treated with the solvent, but at doses 100 and 200 mg/kg/day did not produce a major difference compared with the mice treated with solvent. The mice treated with crude hydromethanolic extract have a lower mean hemoglobin level than mice treated with similar doses of chloroform fraction. The noninfected mice were compared with the treatment group as a customary since earlier peer-reviewed journals used the packed cell volume to gauge anemia associated with P. berghei infection [51]. We used hemoglobin measurements that needed low volume of blood and were easy to research instrumentally in a quick time and compared the packed cell volume between groups.

The three different doses of both the chloroform fraction and crude hydromethanolic extract of *B. antidysenterica* leaves showed an increase in mean survival time compared with mice treated with the solvent, but crude hydromethanolic extract at doses of 100 and 200 mg/kg/day did not produce a major difference compared with the mice treated with solvent. Chloroform fraction at doses of 200 and 400 mg/kg/day showed a significant increase in mean survival time compared with the mice treated with solvent. Significant difference of antimalarial activity was observed in chloroquine-treated mice compared with the mice treated with solvent.

In the curative test, the percent parasitemia level increased from 72 hours to 120 hours in the negative control, and ultimately, all the infected mice died before the sixth day sample was collected. Mice infected with *P. berghei* treated with crude hydromethanolic extract and chloroform fraction of *B. antidysenterica* leaves showed an increase in the percent parasitemia level from day 3 up to day 4 and showed a decrease in percent parasitemia level from day 5 up to day 7 in a dose-dependent manner compared with the mice treated with solvent. The infected mice treated with chloroquine base showed a decrease in average percent parasitemia from 72 hours to 120 hours, and the parasitemia was completely cleared on the 6^th^ and 7^th^ day of treatment.

The promising result from Rane's study suggests that the crude hydromethanolic extract and chloroform fraction of *B. antidysenterica* leaves have therapeutic efficacies against established malarial parasitic infections.

## 5. Conclusion

From this research, we came across a judgment that crude hydromethanolic extract and chloroform fraction of *B. antidysenterica* leaves have shown promising antiplasmodial activity in *P. berghei*-infected mice, which supports its traditional medicine use. Thus, it may be believed to be a possible source to formulate new antimalarial medications; however, these results cannot be applied on to humans due to species variation.

## 6. Recommendation

This research investigated that the plant *B. antidysenterica* leaves have therapeutic values in malarial infections. So, advanced comprehensive studies in *P. falciparum* infection using other appropriate models are needed and justifiable.

*Brucea antidysenterica* is a multipurpose wild plant used for the building of homes, firewood, animal feed, and treatment of various diseases both in humans and other animals that the concerned bodies are advised to require measures to conserve it.

## Figures and Tables

**Figure 1:** Effects of crude hydromethanolic extract and chloroform fraction of *B. antidysenterica* on body weight of *P. berghei*-infected mice in a 4-day chemosuppressive test. *N* = 6, CON = negative control (solvent 10 ml/kg), I = standard error of mean, CM = crude hydromethanolic extract, CF = chloroform fraction of CM, CQ = chloroquine. a, compared with negative control; b, compared with 100 mg/kg; c, compared with 200 mg/kg; d, compared with 400 mg/kg; e, compared with CQ10 mg/kg; f, compared with noninfected mice: 2, *p* < 0.01; 3, *p* < 0.001.

**Figure 2:** Effects of crude methanolic extract and chloroform fraction of *B. antidysenterica* leaves on mean hemoglobin level of mice infected with *P. berghei* in a 4-day suppressive test. *N* = 6, CON = negative control (solvent 10 ml/kg), CM = crude hydromethanolic extract, CF = chloroform fraction of CM, CQ = chloroquine. a, compared with negative control; b, compared with 100 mg/kg; c, compared with 200 mg/kg; d, compared with 400 mg/kg; e, compared with CQ10 mg/kg; f, compared with noninfected mice: 2, *p* < 0.01; 3, *p* < 0.001.

**Figure 3:** Effects of crude hydromethanolic extract and chloroform fraction of *B. antidysenterica* leaves on mean survival time of mice infected with *P. berghei* in a 4-day suppressive test. *N* = 6, CON = negative control (solvent 10 ml/kg), CM = crude hydromethanolic extract, CF = chloroform fraction of CM, CQ = chloroquine. a, compared with negative control; b, compared with 100 mg/kg; c, compared with 200 mg/kg; d, compared with 400 mg/kg; e, compared with CQ10 mg/kg: 2, *p* < 0.01; 3, *p* < 0.001.

**Figure 4:** Effects of crude hydromethanolic extract and chloroform fraction of *B. antidysenterica* leaves on mean survival time of mice infected with *P. berghei* in a suppressive test. *N* = 6, CON = negative control (solvent 10 ml/kg), CM = crude hydromethanolic extract, CF = chloroform fraction of CM, CQ = chloroquine. a, compared with negative control; b, compared with 100 mg/kg; c, compared with 200 mg/kg; d, compared with 400 mg/kg; e, compared with CQ10 mg/kg: 2, *p* < 0.01; 3, *p* < 0.001.

**Table 1:** Preliminary phytochemical screening of hydromethanolic crude extract and chloroform fraction of *B. antidysenterica* leaves.

Phytoconstituents	Type of test	Appearance when positive	Result
Alkaloids	Wagner's and Mayer's tests	Reddish brown and white creamy ppt.	**+**
Anthraquinones	Borntrager's test (chloroform + NaOH)	Red color	−
Cardiac glycosides	Keller–Kiliani test (glacial acetic acid + ferric chloride + concentrated sulfuric acid)	A brown ring	−
Flavonoids	Alkaline reagent test	Colorless	**+**
Phenolic compounds	Ferric chloride	Bluish black	**+**
Resins	Ethanol + distilled water	Formation of a ppt.	−
Saponins	Foam test	Foam	**+**
Sterols	Liebermann–Burchard test (chloroform + acetic acid + sulfuric acid)	Blue green ring	**+**
Tannins	Ferric chloride	A brownish green or blue black coloration	**+**
Terpenoids	Salkowski's test (sulfuric acid + chloroform)	Reddish brown	**+**

+ indicates presence; − indicates absence; ppt.: precipitate.

**Table 2:** Effects of crude hydromethanolic extract and chloroform fraction of *B. antidysenterica* leaves on *P. berghei*-infected mice in a 4-day suppressive test.

Extract	Percent parasitemia	Percent parasitemia inhibition
CON_10 ml/kg_	42.8 ± 1.70	0.00
CM_100 mg.kg_	28.47 ± 0.41^acde(3)^	33.48
CM_200 mg/kg_	17.82 ± 0.39^abde(3)^	58.36
CM_400 mg/kg_	10.3 ± 0.32^abce(3)^	75.93
CF_100 mg/kg_	26.4 ± 0.30^acde(3)^	38.32
CF_200 mg/kg_	15.2 ± 0.73^abde(3)^	64.49
CF_400 mg/kg_	10.00 ± 0.21^abce(3)^	76.64
CQ_10 mg/kg_	0.00 ± 0.00^abcd(3)^	100.00

Data are expressed as mean ± SEM; *n* = 6; CON = control; CM = crude hydromethanolic extract; CF = chloroform fraction of *Brucea antidysenterica*; CQ = chloroquine. a, compared with negative control; b, compared with 100 mg/kg; c, compared with 200 mg/kg; d, compared with 400 mg/kg; e, compared with CQ_10 mg/kg_: 3 = *p* < 0.001.

**Table 3:** Percent parasitemia and percent parasitemia inhibition of *P. berghei*-infected mice treated with crude hydromethanolic extract and chloroform fraction of *B. antidysenterica* leaves in the curative test.

Extract	Day 3 %Para. Supp.	Day 4 %Para. Supp.	Day 5		Day 6 %Para. Supp.	Day 7 %Para. Supp.
			Average percent parasitemia	%Para. Supp.		
CON10 ml/kg	14.10 ± 0.54	34.00 ± 0.83	45.13 ± 0.48	0.00	0.00	0.00
CM100 mg/kg	15.00 ± 0.37	27.03 ± 0.81	24.03 ± 0.68^acd(3)^	46.75	23.07 ± 0.42	18.96 ± 0.78
CM200 mg/kg	14.03 ± 0.60	26.07 ± 0.46	17.10 ± 1.05^abe(3)d2^	62.11	13.27 ± 0.31	10.00 ± 0.47
CM400 mg/kg	15.10 ± 0.18	29.00 ± 0.30	13.13 ± 0.18^abe(3)c2^	70.90	9.07 ± 2.00	7.50 ± 0.17
CF100 mg/kg	12.13 ± 0.20	25.00 ± 0.24	22.43 ± 0.95^acde(3)^	50.30	20.30 ± 0.60	16.40 ± 0.54
CF200 mg/kg	14.05 ± 0.31	20.00 ± 0.52	15.57 ± 0.68^abde(3)^	65.50	11.93 ± 0.72	9.63 ± 0.38
CF400 mg/kg	15.13 ± 0.53	7.07 ± 0.14	9.00 ± 0.15^abce(3)^	80.06	8.70 ± 0.30	7.30 ± 0.33
CQ10 mg/kg	13.10 ± 0.38	34.00 ± 0.83	3.10 ± 0.22^abcd(3)^	93.13	0.00 ± 0.00	0.00 ± 0.00

Data are expressed as mean ± SEM. *n* = 6; CON = negative control; CM = crude hydromethanolic extract, CF = chloroform fraction of *B. antidysenterica*; CQ = chloroquine; % Para. Supp. = percent parasitemia suppression. a, compared with negative control; b, compared with 100 mg/kg; c, compared with 200 mg/kg; d, compared with 400 mg/kg; e, compared with CQ10 mg/kg: 2, *p* < 0.01; 3, *p* < 0.001..

## Data Availability

The data sets used and/or analyzed during the current study are available from the corresponding author and will be delivered to responsible bodies on reasonable request.

## Abbreviations

CQ: Chloroquine
EPHI: Ethiopian Public Health Institute
IC_50_: 50% inhibitory concentration
LD_50_: Median lethal dose 50
PRBCs: Parasitized red blood cells
RBCs: Red blood cells.
